# Optical Microscope Rehabilitation Nursing Study of Anterior Cruciate Ligament Injury through Lateral Knee Incision Based on Medical Internet of Things

This article has been retracted.

**DOI:** 10.1155/2022/1493221

**Published:** 2022-08-16

**Authors:** Liping Liu, Nan Chang, Shihong Li, Peipei Gong, Junhua Wang

**Affiliations:** ^1^Department of Radiology, Jinan Third People's Hospital, Jinan, 250132 Shandong, China; ^2^Department of Respiratory and Critical Care Medicine, Qingdao Municipal Hospital, Qingdao, 266071 Shandong, China; ^3^Department of Hepatobiliary Surgery, Shandong Provincial Hospital Affiliated to Shandong First Medical University, Jinan, 250014 Shandong, China; ^4^Department of Rehabilitation Medicine, Shandong Provincial Hospital Affiliated to Shandong First Medical University, Jinan, 250014 Shandong, China

## Abstract

With the high development of sports, football has attracted more and more attention from the public. However, the hot competition has made football players undergo high-intensity training, and the risk of injury caused by training is also increasing. Lateral incision knee ACL injury is one of the most common types of injuries in football players, which has a serious impact on the athlete's physiology and daily training. The comprehensive, multi-level, convenient and fast medical system brought by the medical Internet of Things has become the growing demand of the medical industry. Based on the medical Internet of Things, this paper studies the rehabilitation nursing of football players' ACL injury by lateral cutting and running combined with optical microscope. In this paper, 36 male and female football players were selected for group experiments, and the landing and peak torque indexes of the experimental group and the control group of male and female athletes were analyzed under the observation of an optical microscope. Group (P <0.05), coxa valgus (P <0.01), internal rotation and knee valgus angles were greater than those in the EM group. And the peak hip flexion angle and knee valgus moment in NF group were lower than those in EF group (P <0.05). After 12 weeks of rehabilitation training, there was a significant difference in the Q/H joint contraction index between the REF group and the CON group (P <0.05), and there was no statistical difference in the other groups. After 12 weeks of rehabilitation training, there was a significant difference in the Q/H joint contraction index between the REF group and the CON group (P <0.05), and there was no statistical difference in the other groups. That is to say, after the systematic rehabilitation training proposed in this paper, the joint contraction performance of the hamstrings/quadriceps in the REF group has been significantly improved. This shows that the rehabilitation nursing under the optical microscope based on the medical Internet of Things has a good effect on the rehabilitation of the football player's side-cut running knee joint ACL injury.

## 1. Introduction

The knee joint is one of the most important structures in the human body. It is the most frequently used and most vulnerable part of the human body. Especially the anterior cruciate ligament injury of the knee joint will seriously affect the human body's standing, balance and other functions, and often associated with meniscus injury, is a high incidence of orthopedic diseases. Especially in the course of sports, the knee joint is often injured due to difficult training and competition. Injuries to the knee joint can have a significant impact on daily activities. After the injury occurs, if it is not treated effectively, it may leave some sequelae, which will seriously affect the physical function of the football player and the daily training.

In some team sports, athletes often have strong physical confrontation capabilities, a variety of sports skills and amazing team spirit. In some team sports competitions, athletes often do such sideways movements. As an important grounding method, the sideways technical movement occupies a very important position in the technical movement training of some specific athletes, especially the most common in group sports such as Football. A large amount of regular sideways technical movement training can easily lead to knee joint injuries, especially anterior cruciate ligament injuries. For this reason, it is of great significance to study the biomechanical properties of football players' knee joints and the rehabilitation theory of anterior cruciate ligament injuries.

Joerg Mika compared the biomechanical characteristics of knee joints for different motor tasks and explored which tasks can cause anterior cruciate ligament injury. Joerg Mika selected 24 female athletes as subjects, and 24 female athletes completed three sports tasks: one-limb landing, implanted amputation, and two-limbed jumping. Joerg Mika calculated the angular displacement of flexion/extension, abduction/adduction and tibial internal and external rotation, and also calculated the angular displacement, abduction and tibial internal rotation. The Joerg Mika study found that during the implantation amputation process In the test, the subject started to touch the tibia, and the tibia rotated faster and turned more deeply into the tibia. The results of Joerg Mika's research show that although one-limb tasks are significantly more likely to cause anterior cruciate ligament injury than bilateral landing, two-limb landings with greater knee abduction may also cause anterior cruciate ligament damage [1, 2]. Pieter Van Dyck compared the biomechanical characteristics of three clinical techniques of anterior cruciate ligament (ACL) -deficient knee joints. Pieter Van Dyck performed three rotation displacement tests (rotation displacement test, jerk test, and N test) on 28 patients with simple anterior cruciate ligament injury. An electromagnetic sensor system was used to evaluate the three-dimensional kinematics of each patient's injured and uninjured knee in each movement. Pieter Van Dyck's results show that the maximum tibial displacement (pCAT) of the pivot shift test is significantly larger than the jerk test and the N test [3].

This article first summarized the relevant theoretical knowledge, made a certain introduction to the knee joint and anterior cruciate ligament, and focuses on the analysis of the biomechanical characteristics of the lateral movement of football. Then 36 subjects were selected for group experiments. A control group experiment was conducted to conduct a study. In the course of the experiment, the joint dynamics parameters, the surface electromyogram of the lateral cut muscle and the co-contraction index of the lower extremity muscles were analyzed experimentally and the relevant conclusions were drawn. In this paper, combined with the medical Internet of Things, the observation under the optical microscope can effectively diagnose the knee joint injury of athletes, provide a new idea for the treatment of sports injury, and provide a new direction for the development of medical intelligence.

## 2. Proposed Method

### 2.1. Knee Joint

#### 2.1.1. Anatomical characteristics of the knee joint

*(1) Knee joint bone*. From the aspect of the articular surface and the bone, the knee joint is composed of the articular surface below the femur, the articular surface above the tibia, and the sacrum, and belongs to the elliptical pulley joint. From the perspective of the support and reinforcement structure of the knee tibial side, the first should be the fascia layer surrounding the outer layer of each muscle group, then the various ligaments attached around the knee joint, and finally the joint capsule of the knee joint [4, 5]. From the perspective of the fibula support and reinforcement structure of the knee joint, the fascia layer should be the first, and then the fibula collateral ligament, and finally the joint capsule of the knee joint. Among them, because the shape of the sub-femoral articular surface and the upper tibial articular surface are not disproportionate, or they are not occluded, there is also a relatively large gap inside the two articular surfaces. Filled with two fibrous cartilaginous plates to match the shape of the upper and lower articular surfaces, thereby increasing the stability of the knee joint, and also can deepen the joint socket to increase the mobility and flexibility of the knee joint. The two fibrocartilage plates are Meniscus [6, 7]. A piece of patellofemoral is surrounded by the quadriceps tendon in front of the femoral block joint, which is mainly to change the tensile line of the quadriceps. Before and after the knee joint, there are also two cruciate ligaments that prevent the mutual movement between the femur and tibia when the knee joint is in a semi-flexed position, resulting in overextension and overflexion of the knee joint, limiting the distance and movement of the tibia forward and backward within the joint Degree, the lateral collateral ligaments on both sides of the knee joint and the lateral collateral ligaments, play a role in preventing excessive knee varus.

*(2) Meniscus*. The meniscus is two fibrocartilage plates inlaid on the articular surface of the tibia and lateral tibial condyle. They are the inner meniscus and the outer meniscus. Among them, the inner meniscus has an approximate letter c shape, and the outer meniscus has an approximate letter o shape. In terms of joint mobility, the lateral meniscus is slightly more active, and the medial meniscus is less active than the lateral meniscus due to its shape and location. The outer and inner edges of the meniscus vary in thickness, with the outer edge being thicker and the inner edge being relatively thin. This helps to reduce the impact of the joint between the head and the socket when the knee is in motion, thereby improving the stability of the knee joint [8]. At the same time, because there is a space around the femoral condyle and tibial condyle around the joint capsule, various ligaments, and periosteum, the meniscus can also cushion the knee flexion and extension in the coronary axis. In addition, the meniscus also helps to strengthen the nutritional supply of cartilage in the joints.

*(3) Knee ligaments*. There are two ligaments in the anterior and posterior part of the knee joint, namely the anterior cruciate ligament and the posterior cruciate ligament. The starting point of the anterior cruciate ligament is located behind the medial side of the lateral femoral condyle. When the knee joint is in flexion, the anterior cruciate ligament has greater tension on the anterior and medial side, and the posterolateral side is relatively loose. When the knee joint flexed about 45 degrees, the anterior cruciate ligament reached its most relaxed moment. At this time, the ligament stress was small and relatively relaxed. The role of anterior cruciate ligament is mainly that, firstly, it restricts the excessive forward movement of the proximal end of the tibia in the knee joint and thus limits the excessive extension of the knee joint. Secondly, the ligaments can also limit the internal rotation and external rotation of the tibia in the knee joint surface, as well as the varus and varus motion of the knee joint in the extended position. The starting point of the posterior cruciate ligament is located behind the lateral surface of the medial condyle of the femur, and the end point is in the sulcus of the tibial intercondylar bulge. Part of the tissue of the posterior cruciate ligament is connected to the lateral meniscus. When the knee joint is in the flexion position, the back of the cruciate ligament is relatively loose and the front is tight. When the knee flexion reaches about 30 degrees, most of the cruciate ligament is in a tight state. Its role is mainly to limit the excessive backward movement of the tibia in the knee joint surface to limit the excessive extension of the knee, but also to limit the internal rotation and external rotation of the knee joint. There are collateral ligaments on both sides of the knee joint. According to their positions, they can be divided into tibial collateral ligaments and fibula collateral ligaments. The tibial collateral ligament is located on the side of the tibia behind the medial knee, the starting point of the ligament is on the medial condyle of the femur, and the stop is on the medial condyle of the tibia. Stretch. The fibular collateral ligament is located on the fibula side behind the lateral knee joint. The starting point of the ligament is located on the lateral femoral condyle and the stop is on the fibula head. The role of the fibula collateral ligament is to fix and limit the knee joint's excessive movement on the coronary axis from the outside. The tibial collateral ligament and the fibular collateral ligament limit and protect the human knee joint, allowing the knee joint to do as much flexion and extension as possible in the coronary axis. Injuries to the knee ligaments can lead to poor joint stability in football players. In severe cases, it can even cause traumatic arthritis and movement disorders in athletes.

#### 2.1.2. Biomechanical characteristics of the knee joint

The knee joint is the most suitable joint for biomechanical analysis. Because although the knee joint movement seems to be only flexion-extension, it is actually one of the most complex joints in the human body with the shoulder joint. The knee joint consists of two joints, the femoro-tibia and patellofemoral joints. The tibiofemoral joint can be divided into medial tibiofemoral joint and lateral tibiofemoral joint. The articular surface of the lateral tibiofemoral joint is irregular. About one-third of the front is a rising concave surface, and about two-thirds of the back is a gradually falling concave surface. The sagittal position of the lateral tibial condyle is an upward convex surface. This plane is related to the anterior segment of the anterior segment of the femur and the posterior segment of the posterior flexion joint. This region is called the lateral tibial articular surface. The medial tibiofemoral joint surface is a bowl-shaped concave surface.

When the knee joint is in the flexed position, the medial tissue of the knee joint is significantly less relaxed than the lateral side, and the same is true when the knee joint is in the extended position. In addition, a small degree of lateral relaxation of the knee joint within a certain range is allowed in knee joint replacement.

For the knee joint, the tibiofemoral surface usually occurs in the tibial condyle and femoral condyle. The facial motion between the tibial condyle and the femoral condyle occurs simultaneously on all three planes, of which the amplitude of motion in the cross section of the human body and the coronal plane is relatively small. Patellofemoral articular surfaces usually occur in the femoral condyles and patella condyles. Between the femoral condyle and the zygomatic condyle, facial movements occur at the same time in the coronal plane and cross section. The range of tibiofemoral joint movement in the coronal plane. When the knee joint moves from full extension to flexion to 30 degrees, the range of adduction or abduction will increase, but no matter what position the knee joint is in the coronal plane Activity is usually only a few degrees.

When the knee joint is fully extended until flexed to a right angle, the joint mobility will increase slightly, but when the knee joint is fully extended, the extent of abduction or adduction is minimal. The tibiofemoral joint has the largest range of joint motion when flexing and extending around the coronary axis. The flexion and extension range can reach 140. The femoral block separates the inner and outer femoral condyles. The femoral block provides a stable sliding track for the patella. There is a pulley groove in the deep part of the pulley, and the angle formed by the pulley groove is normally about 135~140 degrees.

In the patellofemoral joint of the knee joint, the muscle strength of the quadriceps tends to increase as the degree of flexion of the joint increases. From the normal standing state of the human body, the knee joint is continuously flexed. When the knee flexion is increased, the quadriceps muscle strength is continuously increased, and the knee extension torque is continuously increased. At this time, the reaction force of the patellofemoral joint in the knee joint also increased, but in flexion of the knee joint, the patellofemoral joint reaction at any time was greater than the muscle strength of the quadriceps at the same time. The knee joint flexes around the coronary axis until a greater sacral joint reaction occurs when vertical. The reaction force of the patellofemoral joint when vertical can be almost two to three times the gravity of the human body. There is also the case where the knee joint is continuously flexed and the muscle strength of the quadriceps remains unchanged, the reaction force of the patellofemoral joint will still increase.

### 2.2. Anterior Cruciate Ligament of the Knee

#### 2.2.1. Functional anatomy of the anterior cruciate ligament of the knee

The anterior cruciate ligament starts from the medial surface of the lateral femoral condyle [9]. Its approximate length is 31-38 mm, and the average width at the center is 10-12 mm. Its cross-section resembles an oval structure, and there are gender differences. The average area of men and women is 44 mm2 and 36 mm2, respectively. The attachment surface of the anterior cruciate ligament at the end of the tibia is approximately more than three times the cross-sectional area at the midpoint, and it is spread out in a fan-shaped structure at 10.12 mm from the tibial dead center, forming a triangle with a wider anterior side and a narrower side. Or eggs. The circular range has an average sagittal diameter of 17 mm, a coronal diameter of 11 mm, and a total area of 136-150 mm2. The anterior cruciate ligament is at an angle of 30° and 50° on the sagittal plane with the femur and tibia, and is 21° from the femur on the coronal plane. The long axis direction at the femoral dead center is parallel to the direction of the long axis of the femur, and the long axis direction at the tibial dead center is parallel to the direction of the anteroposterior diameter of the tibial plateau. This forms the overall structure that the ACL is rotated around itself. The fiber length of the anterior cruciate ligament is not uniform and there are differences.

From the point of view of the overall structure of the ligament, the posterior outer bundle is located approximately rearward of the anterior inner bundle. This structure determines the tension of the posterior outer bundle when the joint is in a straight state and the anterior inner bundle when the joint is in a flexed state [10]. As the knee flexion angle and tension change, the length of the two bundles will also change accordingly. When the knee joint is at 90° flexion, the length of the outer bundle will decrease by 5-7.1 mm, and the length of the front inner bundle will decrease. Increase 3.3-3.6 mm. Another study suggested that the current cruciate ligament is at 90. When flexed in position and accompanied by inward rotation, its length can increase by 1.7-2.7 mm. The fiber travel of the anterior cruciate ligament is also special. Most of the fiber bundles are distributed along the longitudinal direction, which can limit the forward movement of the tibia and the internal rotation of the knee joint, internal and external turnover, and excessive extension.

Generally, when the quadriceps muscle is strongly contracted, it can drive the knee joint. The anterior cruciate ligament is more stressed when the quadriceps isometrically contracted, and flexion exercises such as squatting and active knee extension are active; the rope muscles also play an important role in the flexion of the knee joint. When the ischial muscle is contracted in equal length and the quadriceps and hamstring muscles are contracted cooperatively, the anterior cruciate ligament bears relatively little stress due to the large flexion angle of the knee joint. In the middle and early stages of the gait cycle (that is, the foot is off the ground), the horizontal shear force on the anterior cruciate ligament is large, especially when one foot leaves the ground, which can produce a maximum stress of about 303 N. During the landing phase of the walking cycle, the force of the anterior cruciate ligament is less because of the contraction of the muscles around the knee joint, the reaction force of the ground with respect to the lower limbs, and the relative force between the tibia and femur. The anterior cruciate ligament is located at the junction of the femur and tibia, with about 1% to 2% of its volume proprioceptors. The central nervous system continuously receives stimulus signals sent by sensor-like proprioceptors. After integration, these proprioceptive signals It continues to be transported from the center to the periphery in the form of vision and vestibular sensation, and the excitability of its corresponding muscle is adjusted by this signal feedback mechanism. The stability of knee movement also requires the joint participation of these mechanisms.

#### 2.2.2. Mechanism of knee anterior cruciate ligament injury

The function of the anterior cruciate ligament depends on its own biological structure and mechanical properties [11]. First, it can counteract the relative movement of the tibia relative to the femur during joint movements, and secondly, it can counteract the forces and rotational forces produced by the varus and knee of the knee joint. When the ligament tissue is subjected to stretching, its structure first produces elastic deformation, and the elastic change ranges from about 7% to 15% of its total length. But no matter how much, as long as the range of change exceeds its maximum value, the ligament will plastically deform or even partially or completely break. Some scholars have measured that the length of the anterior cruciate ligament in China is mostly concentrated around 32 mm. A conservative (i.e. 7% change in length) is used to estimate the elastic range of the ligament. The elastic range of the ligament should be above 2 mm. The force may cause plastic deformation or even fracture of the ligament. In daily life or sports, the anterior cruciate ligament is one of the main movements that cause anterior cruciate ligament injury. In sports such as basketball, football, and skating, some twisting, shearing, and emergency stopping actions are often required. This kind of instantaneous burst force under insufficient preparation can cause great impact on the knee ligaments, especially the anterior cruciate ligament.

#### 2.2.3. Effect of knee joint function after anterior cruciate ligament injury

The knee joint has an irreplaceable role in weight-bearing and maintaining trunk stability. In addition, it is also important for overall exercise. Normal human walking or running requires the cooperation of the knee and hip joints [12]. According to the previous description of the functional anatomy of the knee joint, it can be known that the knee joint does not only perform flexion and extension of a single axial position, it also has two other axial positions, including internal and external rotation and varus. What is more outstanding is that the knee joint can be rotated while doing flexion and extension. According to research, during normal walking, each step of walking is accompanied by two axial movements. The self-protection mechanism of the human body makes the lower limb gait change correspondingly after the current cruciate ligament injury. When the anterior cruciate ligament is completely broken, the stability mechanism of the knee joint is destroyed. Therefore, patients will exercise more careful movements and avoid other actions that may increase discomfort, such as stiff gait. The knee joint can show obvious tibia forward during the squat movement and pivot shift test. This abnormal pattern will also increase knee instability and even cause injury.

### 2.3. Analysis of Biomechanical Characteristics of Football Side Cut

The action that the athlete changes direction during running is called side-cutting action. In the side-cutting movement, the athlete first decelerates in the original direction, one leg stops abruptly, and then the other leg strides in a new direction, that is, a gait that changes direction. The support in the side-cutting gait is the biomechanical characteristics of the stage from the moment when the support leg first touches the ground to the time when the support leg leaves the ground. The maximum flexion angle of the knee joint, which is the time when the angle between the lower leg and the thigh is the smallest, is the boundary point, which is the cushioning stage and the pedaling stage. During the buffering phase, when the human body contacts with external objects, the extensor muscles of the lower limbs perform eccentric contraction to complete the concession work. The cushioning action can reduce the impact of external objects on the human body. When the human body falls from the air, the action transitions through the forefoot to the full foot, bending the ankle, knee, and hip, to reduce the impact of the ground on the human body and prevent lower limb damage. The cushioning action of the lower limbs is mainly to reduce the force between the human body and the moving object, so as to facilitate the control of the object by the human body. The buffering action also provides space and time for the completion of subsequent pedaling and extension actions. At the same time, the extensor muscles are moderately elongated and a certain amount of elastic potential energy is stored, which provides stronger stimulation for the contraction of the extensor muscles and enhances the work efficiency of the muscles during contraction. Stretching is one of the main movements of the lower limbs during the kicking and stretching phase. It is the action process in which the extensor muscles of the lower limbs perform concentric contraction to complete the extension of the lower limbs and exert force on the ground. While stretching the joints, the force on the ground is continuously increased, so that the force on the ground is continuously increased, which makes the human body jump into the air. During the support phase of the sidecut gait, the corresponding biomechanical changes of the hip, knee, and ankle joints will occur.

In the movement of side-cutting movements, due to the characteristics of the movement itself, the shift of the center of gravity during the movement and the changes in the speed and acceleration of the center of gravity change, resulting in changes in the ground reaction force. The force gradually increases and a corresponding peak appears. During the kicking and stretching phase, the center of gravity accelerates due to the kicking and stretching action, causing a second peak of ground reaction force, and then gradually decreases until the foot leaves the ground. The change of ground reaction force will have different effects on the lower limbs. In order to resist the impact of the ground reaction force, the muscles around the joints of the lower limbs will produce different muscle moments. The joint torque is mainly used to control the tension of a joint muscle group, and is the performance of the comprehensive effect of all muscles (including active and antagonistic muscles) across the joint.

## 3. Experiments

### 3.1. Research Object

Based on the medical Internet of Things, this paper conducts a rehabilitation nursing study on the ACL injury of the football player's side-cut running knee under an optical microscope. A total of 36 male and female soccer players were selected as research objects, including 24 females and 12 males. The 36 athletes were divided into: ordinary female athlete group (NF) 10 people; excellent female athlete group (EF) 14 people and excellent male athlete group (EM) 12 people. The EF group was randomly divided into experimental group (REF) Compared with the control group (CON), each group was 7 people. The experimental group received a 12-week rehabilitation intervention and observation therapy using a medical IoT light microscope. The control group was not observed and treated with a light microscope. The value of the general information of the subjects was the mean ± standard deviation (M ± SD) Indicates that the detailed information is shown in Table 1.

Judging from the P value of the judgment hypothesis test results, each index P is less than 0.05. The age, height, weight, years of professional training, and exercise level of each athlete group in this experiment are not significantly different from each other, and there is no history of lower limb pain in the past 6 months or the injuries that affect the completion of this experiment, and no history of knee surgery., And can complete the action according to the experimental design requirements.

### 3.2. Test Steps

#### 3.2.1. Pre-experiment

Four subjects in the normal control group were selected, and side runs were repeated. Three-dimensional motion analysis and SEMG data were collected under light microscope observation. Each subject was tested twice, indicating the repeatability of the experimental instrument test and the reliability of the relevant data. Parameters taken include: peak angles and moments of hip, knee, and ankle joints, joint angles and moments of hip, knee, and ankle at landing, the average RMS of each muscle activity in the test action cycle as a percentage of MVC, and the Contribution rate.

#### 3.2.2. Experimental steps

1. All the athletes undergo clinical examination and diagnosis to rule out experimental contraindications. Started synchronous testing of 3D motion analysis system and EMG test system. Observe the kinematics, dynamics indexes, and myoelectricity indexes of the dominant side joints of each group
2. The EF group was divided into the CON group and the REF group, and a preventive rehabilitation training program was implemented for the REF group, without intervention in the CON group. Both groups did not affect routine training, and all rehabilitation interventions were conducted under the guidance of team doctors, four times a week, interspersed with daily training. After 12 weeks, the clinical evaluation and experimental tests were repeated for the athletes in the CON and REF groups. To observe the effects of the rehabilitation training program on the kinematics and dynamics of the dominant side of the lower limbs and the SEMG of the main muscles around the knee joints
3. Intervention plan: Select the PEP injury preventive rehabilitation fitness training program, frequency: 4 times a week for a total of 12 weeks. All training content is completed under the guidance of team doctors, combined with balance ability training

### 3.3. Data Analysis

All statistical analyses were performed using the SPSS22.0 software package. The parameters of the REF group and the CON group before and after the rehabilitation training were compared by single factor analysis of variance (ANOVA). The parameters of the EF group, the EM group, and the NEF group were compared using the independent sample t test. P <0.05 indicates that the data comparison has Significant difference, P <0.01 indicates that the data comparison has a very significant difference. Normal distribution measurement data is expressed by (x ± s). Two samples are compared using the independent sample t-test when homogeneity of variance is used.

## 4. Experimental Results and Analysis

### 4.1. Analysis of Articulation Parameters of Soccer Players

#### 4.1.1. Comparison of peak dynamic parameters of lower limb joints between male and female soccer players

The comparison of the peak parameters of the lower limb joint dynamics of male and female soccer players is shown in Table 2.

From the data in Table 2, it can be seen that the athletes in the EF group and the EM group have significant differences in the technical movements in completing the side cut. <0.05), and there is a very significant difference in the peak flexion moment of the hip joint (P <0.01), and there is no significant difference in the related data of the knee joint. That is, the peak flexion angle of female hip athletes at the time of completing the lateral cut is smaller than that of male olive athletes, and the angle of hip inversion and internal rotation is also significantly larger than that of male athletes.

#### 4.1.2. Comparison of kinematic parameters of men and women soccer players at the moment of landing

Table 3 shows the comparison of the kinematic parameters of men and women soccer players at the time of landing.

From the data in Table 3, it can be seen that there is a significant difference between the flexion angle of the hip joint and the flexion moment of the hip joint at the moment of landing when the EF group and the EM group complete the lateral cut (P <0.05). The very significant difference (P <0.01) was that the female flexion and internal rotation angles of the female athletes were significantly larger than those of the EM group, and the knee flexion angles were smaller than those of the male athletes.

### 4.2. SEMG Analysis of Soccer Players' Lateral Running Muscles

#### 4.2.1. Comparison of the muscle contribution rate of the male and female athletes in the lateral cut

In this article's side running movement, each muscle contribution rate is the percentage of each muscle integral electromyogram value to the total value of 7 measured muscles. The comparison of the muscle contribution rate of male and female athletes in side running is shown in Figure 1.

As can be seen from Figure 1, in the EF group athletes' lateral cut test, the median femoral muscle contributed the highest and the gastrocnemius lateral head contributed the lowest. The EM group completed the test movement support phase. The median hamstring muscle contributed the highest and the gastrocnemius lateral head contributed the lowest.

#### 4.2.2. Comparison of Muscle Contribution Rates of Female Olive Athletes in Different Levels

The comparison of the muscle contribution rate of female olive athletes in different levels of side running is shown in Figure 2.

It can be seen from Figure 2 that in the sidecut test of ordinary female soccer players, the median femoral muscle has the highest contribution rate and the gastrocnemius lateral head has the lowest contribution rate. The EF group is ranked according to the contribution rate: medial femoral muscle, medial hamstring muscle, medial head of gastrocnemius muscle, medial hamstring muscle, lateral femoral muscle, rectus femoris, and lateral head of gastrocnemius muscle. Women's soccer players have the same muscle contribution rate in the same order. During the support phase, the muscle contribution rate of the EF group and the NF group is relatively consistent, and there is no significant difference in the contribution rate between the muscle groups (P >0.05).

#### 4.2.3. Comparison of the muscle contribution rate of female olive athletes in the lateral cut before and after preventive rehabilitation training

Figure 3 shows the comparison of the muscle contribution rate of female olive athletes in the lateral cut before and after preventive rehabilitation training.

It can be seen from Figure 3 that after 12 weeks of targeted rehabilitation training, during the cycle of the sidecut running, the contribution rate of each muscle group of the athlete has changed, that is, the medial femoral muscle of the REF group before and after rehabilitation training. The proportion of contribution rate was significantly reduced (P <0.05), while the contribution rate of the hamstring muscle on the back of the knee joint was significantly increased. Through rehabilitation training, the muscle group contribution rate of the REF group changed, with the highest contribution rate of the medial hamstring and the lowest contribution rate of the lateral head of the gastrocnemius. After the rehabilitation training, in the side cut running test of female soccer players, the order of the median hamstring muscle, medial femoral muscle, medial gastrocnemius muscle, lateral hamstring muscle, lateral femoral muscle, rectus femoris, lateral gastrocnemius muscle is ranked according to the contribution rate.

### 4.3. Analysis of Common Contraction Index of Lower Limb Muscles in Soccer Players

#### 4.3.1. Comparison of the Common Muscle Contraction Index (CI) of Lower Limb Muscles for Men and Women soccer players

Table 4 compares the common muscle contraction index (CI) of the lower limb muscles of male and female soccer players.

As can be seen from Table 4, there was a significant difference in the H/Q and LG/LH co-contraction indices between the EF group and the EM group (P <0.05). The hamstring/quadriceps (H/Q), The gastrocnemius lateral head/lateral hamstring muscle (LG/LH) co-contraction performance was higher than the EF group.

#### 4.3.2. Comparison of muscle contraction index of female olive athletes before and after preventive rehabilitation training

Figure 4 show the comparison results of muscle contraction index of female olive athletes before and after preventive rehabilitation training.

It can be seen from Figure 4 that after 12 weeks of rehabilitation training, there was a significant difference in the Q/H co-contraction index between the REF group and the CON group (P <0.05), and there was no significant difference in the other groups. That is to say, System rehabilitation training after observation of optical microscope under medical Internet of Things, the common contractility of the hamstrings/quadriceps muscles of the REF group has improved significantly.

#### 4.3.3. Comparison of body fat percentage and muscle mass

Figures 5 and 6 show the changes in body fat percentage and muscle mass in female soccer players before and after preventive rehabilitation training.

From Figure 5, we can see that before and after the rehabilitation training, the body fat rate of the athletes decreased significantly. The decrease in the fat rate means that the subcutaneous tissue fat of the athletes decreased after the rehabilitation training, and the body became stronger. This shows that rehabilitation training has a certain effect on restoring the physiological function of football players.

As can be seen from Figure 6, after 12 weeks of rehabilitation training, the female athletes have significantly increased muscle weight while the body fat percentage has decreased. It shows that the rehabilitation training method proposed in this paper has obvious effect on the muscle growth of athletes.

## 5. Conclusions

Sports injury is a problem often encountered during exercise. A report released by the American Professional Sports League shows that Football sports ranks second in injury risk in the world's popular sports, and the knee joint has the highest risk of injury relative to other parts of the body. Anterior cruciate ligament (ACL) injury is one of the serious sports injuries common in football players during the game. Anterior cruciate injury can seriously affect athletes' sports performance and quality of life. To this end, this paper raises the research on the biomechanical characteristics of knee joints of soccer players and the rehabilitation theory of ACL injury.

This article conducts research by setting up control experiments. In this paper, under the light microscope, we found that among female athletes of different levels, we found that the vastus lateralis had the highest contribution rate and the lateral head of the gastrocnemius had the highest contribution rate. The medial femoral muscle, as the main muscle of the anterior group of the lower limbs of the human body, plays this important supporting role during the exercise phase.

The results of this study show that football players of different genders and levels have obvious biomechanical risk factors during the side cutting action cycle, and emphasize the importance of optical microscopy based on the medical Internet of things for the rehabilitation of football players' side cutting knee ACL injuries. Restoring normal lower extremity muscle balance and overall lower extremity neuromuscular function is an important principle for soccer players in preventing ACL injury. In addition, there are still many deficiencies in this research work. For example, the actual injury rate lacks long-term efficacy observations. The relevant indicators selected in this article may not fully reflect the biomechanical characteristics of athletes and the clinical effects of preventive rehabilitation training. These deficiencies will be continuously improved in future research work, and the light microscope rehabilitation treatment under the medical Internet of Things will be better integrated with the anterior cruciate ligament injury of football players, providing more realistic research.

## Figures and Tables

**Figure 1:** Comparison of muscle contribution rate between EF group and EM group.

**Figure 2:** Comparison of muscle contribution rate between EF group and NF group.

**Figure 3:** Comparison of muscle contribution rate between CON group and ref group after rehabilitation training.

**Figure 4:** Comparison of the common contraction index of different muscle groups of female olive athletes before and after rehabilitation training.

**Figure 5:** Changes in body fat percentage of athletes.

**Figure 6:** Changes in Muscle Weight in Athletes.

**Table 1:** General data of subjects (M ± SD).

Index	Group NF (N =10)	Group EF (N =14)	Group EM (N =12)	Group REF (N =7)	Group CON (N =7)
Age (years)	21.4 ± 1.4	18.1 ± 1.3	17.4 ± 1.2	18.0 ± 1.4	16.8 ± 0.8
Height (cm)	172 ± 4.2	173 ± 3.8	184 ± 4.1	173 ± 5.2	173 ± 3.1
Weight (kg)	64.7 ± 3.5	65.3 ± 3.1	83.2 ± 4.0	63.3 ± 3.9	63.2 ± 4.4
Years of professional training	6.5 ± 1.7	8.8 ± 1.2	8.7 ± 1.2	9.0 ± 1.4	8.5 ± 1.0

**Table 2:** Peak value comparison of dynamic parameters of joints of elite male and female soccer players (M ± SD).

		EF(N =14)	EM(N =12)	P
Coxa coronal plane	Entropion/valgus	-13.26 ± 8.27	-8.76 ± 5.83	0.042
	Moment	1.91 ± 1.04	1.41 ± 0.33	0.547
Sagittal plane of hip	Flexion/extension	47.35 ± 7.67	59.35 ± 10.91	0.021
	Moment	1.61 ± 0.26	3.18 ± 0.52	0.021
Frontal surface of hip	Internal/external rotation	11.01 ± 6.67	6.23 ± 4.79	0.013
	Moment	-1.03 ± 0.18	-1.02 ± 0.21	0.879
Coronal plane of knee	Extension/back extension	26.2 ± 6.68	27.19 ± 5.73	0.903
	Peak torque	3.81 ± 1.01	3.72 ± 1.12	0.9385
Sagittal plane of knee	Entropion/valgus	4.32 ± 7.08	5.23 ± 7.84	0.416
	Peak torque	0.95 ± 0.92	0.87 ± 0.89	0.815
Frontal surface of knee	Internal/external rotation	6.15 ± 7.78	8.23 ± 6.19	0.475
	Peak torque	0.57 ± 0.01	0.59 ± 0.01	0.974

**Table 3:** Comparison results of kinematic parameters of male and female soccer players at landing time (M ± SD).

		EF(N =14)	EM(N =12)	P
Coxa coronal plane	Entropion/valgus	-4.36 ± 1.27	-3.96 ± 1.83	0.448
	Moment	0.14 ± 0.14	0.22 ± 0.13	0.537
Sagittal plane of hip	Flexion/extension	44.8 ± 6.69	59.35 ± 7.91	0.042
	Moment	-0.56 ± 0.16	-1.08 ± 0.06	0.022
Frontal surface of hip	Internal/external rotation	11.01 ± 6.67	6.13 ± 4.79	0.037
	Moment	0.23 ± 0.18	0.22 ± 0.21	0.973
Coronal plane of knee	Extension/back extension	6.2 ± 1.68	12.19 ± 5.73	0.000
	Peak torque	0.12 ± 0.01	0.09 ± 0.02	0.659
Sagittal plane of knee	Entropion/valgus	21.32 ± 7.08	19.83 ± 7.84	0.845
	Peak torque	0.31 ± 0.12	0.29 ± 0.10	0.891
Frontal surface of knee	Internal/external rotation	6.15 ± 3.78	7.93 ± 3.19	0.478
	Peak torque	0.52 ± 0.32	0.52 ± 0.30	0.939

**Table 4:** Comparison of the common contraction index of each muscle group of the elite male and female soccer players (M ± SD).

Co contraction index(CI)	Grouping	M ± SD	P
GM/MH	EF	1.21 ± 0.87	0.36
	EM	1.58 ± 0.45	
LG/LH	EF	1.50 ± 0.91	0.047
	EM	2.07 ± 1.41	
HQ	EF	0.32 ± 0.17	0.043
	EM	0.58 ± 0.23	
VL/LH	EF	2.47 ± 1.13	0.764
	EM	2.29 ± 1.07	

## Data Availability

No data were used to support this study.
